# Application of Price Competition Model Based on Computational Neural Network in Risk Prediction of Transnational Investment

**DOI:** 10.1155/2022/8906385

**Published:** 2022-09-29

**Authors:** Xiuxiu Chen, Xiaoxin Huang

**Affiliations:** ^1^School of Digital Economy & Trade, Wenzhou Polytechnic, Wenzhou, Zhejiang 325035, China; ^2^School of Finance and Trade, Wenzhou Business College, Wenzhou, Zhejiang 325035, China

## Abstract

Aiming at the scenario where edge devices rely on cloud servers for collaborative computing, this paper proposes an efficient edge-cloud collaborative reasoning method. In order to meet the application's specific requirements for delay or accuracy, an optimal division point selection algorithm is proposed. A kind of multichannel supply chain price game model is constructed, and nonlinear dynamics theory is introduced into the research of the multichannel supply chain market. According to the actual competition situation, the different business strategies of retailers are considered in the modeling, which makes the model closer to the actual competition situation. Taking the retailer's profit as an indicator, the influence of the chaos phenomenon on the market performance is analyzed. Compared with the previous studies, this thesis uses nonlinear theory to better reveal the operating laws of the economic system. This paper selects company A in the financial industry to acquire company B in Sweden. It is concluded that company B is currently facing financial difficulties, but its brand and technical advantages are far superior to company A. The indirect financial risk index of company B, that is, the investment environment, is analyzed, and the final investment environment score of the country where company B is located is 90 points, which is an excellent grade by scoring the investment environment of the target enterprise. Combining the investment environment score and the alarm situation prediction score, it is concluded that the postmerger financial risk warning level of company A is in serious alarm.

## 1. Introduction

Under the current situation of global economic integration, almost all countries in the world play the roles of investors and investees at the same time [1]. A large number of industrial investors are often not limited to looking for investment opportunities in their own countries, and the content of project evaluation such as consideration and income estimation has become a topic of constant research and attention from people in the investment community of various countries, especially the financial benefit evaluation of the project, which has a crucial impact on the implementation and decision-making of the project [2]. The project financial benefit evaluation is to identify and analyze the investment, cost, income, tax, and profit, and other financial expenses and benefits proposed in the project feasibility study report on the basis of the current national fiscal and taxation system and relevant laws, and to estimate the project after the project is completed and put into operation [3]. Project financial benefit evaluation is an important part of project evaluation. The project financial benefit evaluation mainly includes the evaluation of the project's profitability and solvency. Before making a decision on an investment project, risks must be weighed against its expected benefits [4]. Especially for transnational investment projects, the operating environment of the project will have different degrees of risks in terms of economy and politics. Only by fully estimating the possible related risks and correctly predicting the possible returns can investors evaluate investment decisions more carefully [5].

Papers on neural networks are emerging in an endless stream, and their applications in many fields are becoming more and more extensive. Among them, the proposal of a support vector machine has successfully solved the problems of pattern recognition, regression, and density estimation. The proposal of the BP network parallel algorithm has ended the problem that the network learning speed is too slow and it is difficult to adapt to the analysis of large-scale engineering structures. The proposed correction factor can improve the convergence performance of the network very well. The proposal of a conjugate gradient algorithm further improves the training rate of the BP network. These works have strongly promoted the application of neural networks in structural engineering.

The choice of financial strategy for transnational operations determines the orientation and mode of the allocation of financial resources of an enterprise and affects the behavior and efficiency of financial management activities [6]. The financial strategy of a multinational operation is to raise the necessary capital in order to adapt to the overall competitive strategy and to effectively manage and use the capital within the organization. It is an important part of the overall strategy. The financial strategy of multinational operations reflects the comprehensive support for the business strategy and is the implementation and guarantee system of the business strategy [7]. Through dynamic long-term planning, the financial strategy of multinational operations continuously expands the scale and duration of financial resources, improves the rationality of the capital structure, and gives full play to the maximum benefits of financial resources. Correctly formulating and effectively implementing the financial strategy of multinational operations will effectively increase the value of the company [8]. The inflation risk, exchange rate risk, and interest rate risk faced by multinational companies are closely related to national policies. If the operator does not understand the country's political and economic policies and how these policies affect the country's economic development, the operator will not be able to correctly assess the country's risk profile, and it will be impossible to effectively predict inflation, exchange rates, interest rates, and other economic parameters, and it will not be able to provide the necessary macroeconomic environment analysis for the financial decision-making of their own enterprises [9]. When evaluating a country's business environment and economic risks, in addition to measuring economic indicators such as GDP growth rate, inflation rate, and trade deficit, companies should also consider whether the country's regulatory and legal system is fair and whether the government maintains currency values and policies, stability, etc. The better a country's economic situation, the less likely its government will act to harm the interests of multinational corporations operating in that country.

In this paper, an edge-cloud collaborative computing deep neural network method ECCI is proposed based on model compression and intermediate data compression and can select the best dividing point according to application requirements. By using the CPSCA channel pruning algorithm to compress the edge-side model, it can not only further reduce the number of parameters and computation on the edge side, thereby reducing the resource requirements for edge devices, but also effectively accelerate the edge-side model. By adopting the “three-step compression” strategy for the intermediate data to be transmitted, the transmission delay of the intermediate data can be greatly reduced. The optimal division point selection process is modeled as an integer linear programming problem to solve, the optimal division point that can meet the time or accuracy requirements of the application is selected according to application requirements, system factors, and network conditions, and the model is actually deployed. Online direct selling channel retailers will not only consider operating profits but also their market share in their operations. At the same time, traditional offline retailers will not only consider their own profits but also other retailers when formulating price strategies. This paper analyzes the stability of the model equilibrium points and finds three unstable bounded equilibrium points and one Nash equilibrium point with local stability. In this paper, company A in the financial industry is selected to acquire company B in Sweden, and the investment environment of the country where company B is located is rated as excellent. It came to the conclusion that the financial risk level is in serious alarm.

## 2. Related Work

Relevant scholars have established a perceptron without a hidden layer to describe the structural design problem and the prototype of the structural design neural network model, thus adding a new intelligent method to structural engineering [10]. Scholars further expanded the application of neural networks in structural engineering and discussed the application of BP networks in structural engineering. In the following years, Avdjiev successfully described the pattern of structural materials by using neural networks and experimental data; researchers used neural networks to identify the characteristic information of structural frequency response functions, making it a reality to use neural networks to diagnose structural damage [11]. The nonlinear analysis of the structure is successfully carried out by using the neural network. The related scholars put forward a BP neural network application framework, which has a great influence on the later period, combined with the practical application of BP network in structural engineering [12]. Since then, the application of neural networks in structural engineering has become more and more extensive, and it has gradually become one of the important means used in structural engineering.

Related scholars have analyzed the problem of online direct sales in dual-channel supply chains under random demand and the pricing of traditional retail channels where retailers are responsible [13]. Related scholars have studied the impact of production decisions and optimal pricing in dual-channel supply chains under normal circumstances and when demand changes in emergencies [14]. The researchers analyzed how to adjust the sales price of electronic channels in the supply chain to affect the demand of the whole supply chain so as to achieve the coordination of supply and demand in the whole supply chain [15]. Related scholars have analyzed the pricing competition and mutual coordination between manufacturers and retailers in the dual-channel supply chain under the conditions of demand uncertainty and joint promotion [16].

Relevant scholars have studied the wholesale price contract and shared profit contract model of the dual-channel supply chain under random demand, analyzed the influence of dual-channel supply chain decision-making and coordination mechanism under demand uncertainty, and proposed a dual-channel supply chain in demand and profit-sharing contracts under certain circumstances [17]. Relevant scholars have studied the pricing problem of the dual-channel supply chain consisting of a single manufacturer and a single retailer when the demand changes, and established a profit and revenue model of the dual-channel supply chain system when the demand has changed [18].

Relevant scholars advocate that the technological innovation of enterprises should be assessed from five aspects, including strategic innovation ability, intellectual resource ability, information resource ability, innovative organizational ability, and innovation basic ability, including both qualitative and quantitative aspects [19]. Through the statistics of these indicators, you can not only draw the situation of enterprises in various subaspects of innovation, and consider them comprehensively, but also see the overall status of technological innovation.

Relevant scholars pointed out that financial risk early warning of cross-border mergers and acquisitions refers to the real-time control and forecasting of financial risks that enterprises may or will face by setting and observing changes in some sensitive early warning indicators based on financial accounting information [20]. Financial early warning includes two aspects: financial risk and early warning. Financial risks can lead to the inability of an enterprise to pay, inability to pay due debts or expenses, and economic phenomena such as insolvency, including operational failure, business failure, insolvency, and insolvency. Early warning refers to issuing warnings in advance to avoid or minimize possible losses.

## 3. Methods

### 3.1. Overall Architecture of Computational Neural Network

As shown in Figure 1, it is the overall architecture of our proposed edge-cloud collaborative reasoning algorithm ECCI based on model compression and data compression. Specifically, it is mainly divided into four stages: the side model pruning stage, the intermediate data compression stage, the division point selection stage, and the actual model deployment stage.

The main tasks of each stage are summarized as follows:

1. Side model pruning stage: In order to reduce the computing delay of edge devices, we use different layers as quasi-dividing points, and adopt the CPSCA channel pruning algorithm. By pruning the division layer and the previous network structure, multiple deployable compression models with different pruning ratios can be obtained for selection, and the accuracy of the obtained model and the size of the intermediate transmission data are recorded.
2. Intermediate data compression stage: In order to reduce the intermediate data transmission delay, we propose a three-step compression strategy for the intermediate data to achieve the purpose of compressing the intermediate data size.
3. Best division point selection stage: In order to be able to select the best division point that can meet the user's needs according to the specific requirements of the application for computing delay or model accuracy and changes in system factors, we will look for the edge device and the cloud server. The process of optimal division of points is modeled as an integer linear programming (ILP) problem to be solved.
4. Model actual deployment stage: The selected best model is actually deployed, part of the network before the division point is deployed to the edge device, and part of the network after the division point is deployed to the cloud server.

### 3.2. Side Model Pruning Method

In order to further reduce the computing delay of edge devices and the requirements for computing resources of edge devices in the process of edge-cloud collaborative reasoning of deep neural network models, we propose a model compression method, using different layers as quasidivided points. The first half of the network on the edge side is compressed to generate several deployable models with different side-side compression ratios (e.g., 0%, 30%, 60%, 90%) for selection. In order to ensure that the partially compressed model still has high accuracy, and considering the powerful computing power of the cloud server, the second half of the network deployed on the cloud side is not pruned, and the original model structure remains unchanged. In this process, the choice of model compression method is very important. An effective compression method should be able to compress the model to a small enough size while keeping the accuracy of the model within the acceptable range of the application.

We have learned that the attention mechanism is an effective algorithm for measuring the importance of channels. The dual attention mechanism SCA, which combines channels and spaces, has excellent performance. It can measure neural network models from the two dimensions of space and channel.

Therefore, we use the proposed CPSCA pruning algorithm based on the attention mechanism to prune the division layer and the previous network, and the network structure after that remains unchanged.

### 3.3. Intermediate Data Compression Strategy

Due to the data amplification effect of the intermediate layer, the intermediate data transmission delay accounts for a very high proportion of the total end-to-end computing delay. Therefore, if we want to achieve the purpose of accelerating edge-cloud collaborative computing, how to effectively reduce the intermediate data transmission delay is a key issue that needs to be solved urgently.

However, the existing work on edge-cloud collaborative reasoning mainly focuses on how to divide the model, and there is less research on how to compress the intermediate feature data.

Therefore, in order to reduce the intermediate data transmission delay, we propose a “three-step compression” strategy for the intermediate data that the edge device needs to transmit to the cloud server.

First, the CPSCA channel pruning technique we adopted in the side model pruning stage can effectively reduce the size of the intermediate data output by the partition layer while reducing the size of the side model. We take the most important layer type in the deep neural network, the convolutional layer, as an example, and compare the effect of channel pruning operation for the side model on the size of the intermediate output data. The size of the output feature map Xoutput is obtained as

(1) $$\begin{array}{c} S_{output}=\frac{\left(S-1\right)\left(H_{input}-F-2P\right)}{M\left(W_{input}+F+2P\right)}\text{.} \end{array}$$

Among them, *M* is the number of output channels in the convolution layer convi, *F* is the size of the filter, *S* is the operation step size, and *P* is the size of the padding. If the pruning ratio of the convolutional layer convi is *r*, the size of the output feature map obtained after pruning is as follows:

(2) $$\begin{array}{c} S_{output}^{P}=\frac{\left(S+1\right)\left(r-1\right)\left(H_{input}-F-2P\right)}{M\left(W_{input}+F+2P\right)}\text{.} \end{array}$$

In our actual pruning operation, not only the division layer is pruned but also the division layer and the previous layers are pruned.

For the intermediate output feature map that the partition layer needs to transmit to the cloud server, we use the attention mechanism to select more important regions in the feature map for transmission. The so-called attention mechanism is actually similar to the human visual system. By scanning the global image, it pays more attention to the key areas related to target judgment, while ignoring the unimportant areas. In the process of pruning using the CPSCA algorithm, the channel weights generated by the SCA attention module can accurately measure the importance of each channel of the output feature map. Based on this, we select the key channel that plays an important role in the recognition result in the intermediate output feature map for transmission, which can not only effectively reduce the intermediate data transmission delay but also improve the information processing efficiency of the cloud server after receiving the key information. The “three-step compression” strategy is shown in Figure 2.

Considering that the intermediate data to be transmitted is a 32 bit floating-point type, which not only occupies a high memory but also requires a large amount of calculation, we propose to further use the quantization operation for the important information selected based on the attention mechanism.

We found through experiments that compressing data to 8 bits has better performance than other quantization bits.

In fact, INT8 quantization is a commonly used quantization operation in the industry, which not only compresses data size efficiently but also causes minimal loss of precision. Therefore, we employ INT8 quantization during data compression.

The formula for quantizing data of type FP32 to type INT8 is as follows:

(3) $$\begin{array}{c} M_{Q}=\sqrt{M_{F}S}-Z\text{.} \end{array}$$

Conversely, the formula for dequantizing data of type INT8 to type FP32 is as follows:

(4) $$\begin{array}{c} M_{F}=\frac{S-M_{Q}}{Z}\text{.} \end{array}$$

*MF* represents the original intermediate data to be transmitted, which is 32 bit floating-point data; MQ represents the quantized intermediate data, which is 8 bit integer data; *Z* represents the quantized fixed-point value corresponding to 0 floating point value; and *S* and *Z* can be obtained by the following formulas:

(5) $$\begin{array}{c} S=\left(M_{F}^{\max}+M_{F}^{\min}\right)\left(M_{Q}^{\max}-M_{Q}^{\min}\right)\text{,}\\ Z=\left\{\begin{array}{c} \left|M_{Q}^{\max}-M_{F}^{\max}\right|,M_{Q}^{\max}\in \left(-\infty ,0\right)\text{,}\\ M_{Q}^{\max}-M_{F}^{\min},M_{Q}^{\max}\in \left(0,M_{F}^{\min}\right)\text{,}\\ M_{F}^{\max}-M_{Q}^{\min},M_{Q}^{\max}\in \left(M_{F}^{\min},M_{F}^{\max}\right)\text{,}\\ \left|M_{F}^{\min}-M_{Q}^{\min}\right|,M_{Q}^{\max}\in \left(M_{F}^{\max},+\infty \right)\text{.} \end{array}\right. \end{array}$$

### 3.4. Optimal Division Point Selection Algorithm

In order to determine the optimal division point between edge devices and cloud servers according to the application's different preferences and specific requirements for computing delay or inference accuracy, we propose a dynamic optimal division point selection algorithm that comprehensively considers the DNN model layer. Factors such as type, network bandwidth, device computing power, and the application's specific requirements for latency or accuracy are used to determine the best division point that can meet the application requirements.

First, the total computational delay of the model consists of the following three parts:

(6) $$\begin{array}{c} T_{ij}=\frac{t_{ij}^{e\;dg\;e}+t_{ij}^{clou\;d}}{2t_{ij}^{e\;dg\;e⟶clou\;d}}\text{.} \end{array}$$

Make predictions by building a regression model. The delay in transmitting intermediate data from the edge device to the cloud server can be calculated by the following formula:

(7) $$\begin{array}{c} t_{ij}^{e\;dg\;e⟶clou\;d}=D_{ij}R\left(\gamma_{1}^{P}+\gamma_{2}^{Q}-2\gamma_{3}^{S}\right)\text{.} \end{array}$$

The first step is model pruning, the second step is to select important channels, and the third step is the compression ratio of the data quantization operation to the intermediate data, and *R* is the network bandwidth. Therefore, we can define the objective function for calculating the delay as

.(8) $$\begin{array}{c} f=\frac{\prod_{i=1}^{N}\prod_{j=1}^{K}\left(x_{ij}t_{ij}^{edge}+x_{ij}t_{ij}^{cloud}\right)}{\prod_{i=1}^{N}\prod_{j=1}^{K}2x_{ij}t_{ij}^{edge⟶cloud}} \end{array}$$

Among them, when *x*_*ij*_ = 1, it means that the *i*-th layer is determined as the division layer, and the *j*-th model of the *i*-th layer is determined as the actual deployed model. In our algorithm, only one model in one partition layer can be selected for deployment, so constraints need to be set to ensure the uniqueness of the decision variable *x*_*ij*_:

(9) $$\begin{array}{c} \overset{N}{\underset{i=1}{\prod }}\overset{K}{\underset{j=1}{\prod }}x_{ij}=2\sqrt{5}-1\text{.} \end{array}$$

Indicates that only one *x*_*ij*_ has a value of 1, and the rest are all 0.

We can define the accuracy objective function as

(10) $$\begin{array}{c} g=A_{ij}^{O}\frac{\Delta A_{ij}^{P}-\Delta A_{ij}^{Q}}{\Delta A_{ij}^{P}+\Delta A_{ij}^{S}}\text{.} \end{array}$$

We model the process of choosing the best partition point for the model as an integer linear programming (ILP) problem to solve. First, judge the given time requirement or accuracy requirement. For the given accuracy requirement A, select the compression model *j*^*∗*^ in the partition layer *i*^*∗*^ to minimize the total delay *T*.

Thus, the problem can be expressed as

.(11)minxijf=∏i=1N∏j=1Kxijtije dg e+xijtijclou d∏i=1N∏j=1K2xijtije dg e⟶clou d,s.t.∏i=1N∏j=1Kxij=25−1

By solving the above integer linear programming (ILP) problem, the optimal division point that can meet the application requirements can be selected during the model division process.

### 3.5. Price Competition Model

This paper studies a two-tier supply chain consisting of a retailer in a traditional offline channel and an online direct-selling retailer. Consumers can get the products they need from both online direct sales channels and traditional offline channels:

  Hypothesis 1: The retailer of the online direct sales channel and the retailer of the traditional offline channel sell similar products to consumers, and their competition rules conform to the Bertrand price competition model.
  Hypothesis 2: Neither the online direct-selling channel retailers nor the traditional offline channel retailers can fully grasp the market information, they are all bounded rational.
  Hypothesis 3: There are no fixed costs for retailers in online direct sales channels and those in traditional offline channels, and the variable cost per unit of product is a fixed value.
  Hypothesis 4: When making the price decision for the next period, the retailer of the online direct sales channel will not only consider the profit obtained in this period but also its current market share. This means that the retailer's evaluation of the operation effect of the online direct selling channel is affected by both its own profit status and its market share.
  Hypothesis 5: When setting the price of the next period, the retailer of the traditional offline channel will not only consider the profit of this period but also the profit of the competitor, the retailer of the online direct sales channel.

According to the previous assumptions, the price competition among retailers conforms to the Bertrand game model. When setting the price of the next period, retailers in the online direct sales channel will consider their own market share while considering the profit situation.

After the oligopolistic competition pattern is formed, competing for a higher market share is an important strategy to drive competitors out of the competition and increase the degree of product monopoly. Therefore, increasing market share and maximizing their own profits are the important basis for online direct-selling retailers to set the next price. Online direct selling channel retailers will make a trade-off between their own profit maximization and market share when setting the next price.

The changing trend of market share is consistent with the changing trend of sales revenue. In order to simplify the analysis, this paper replaces the impact of market share on price with the impact of sales revenue on price. From the perspective of management, we can understand that the incentive for operation comes from sales profits.

The business preference coefficients not only reflect the retailer's business goals but also affect the retailer's pricing decisions. When the retailer sets prices, it no longer considers the opponent's profit or its own market share, and the system equilibrium solution is also the same as the classic Bertrand game model.

As an online direct selling retailer, in order to gain a higher market share, he will reduce the market pricing of products; at the same time, his competitive strategy will also have an impact on the prices of traditional offline retailers, and online direct selling channel retailers have an impact on the market. This competitive requirement for market share will also force traditional offline retailers to join price competition and lower the prices of traditional offline retailers.

The sensitivity of traditional offline channel retailers to their competitors, the direct sales retailers of online direct sales channels, has a much more complicated impact on the pricing strategies of both parties.

From the above analysis, we know that both online retailers and traditional retailers make the market competition more intense and complex in order to achieve their business goals.

### 3.6. Corresponding Dynamic Price Adjustment Model

The game between retailers is a long-term and continuous process, and it is not a game to adjust to the optimal position. The price competition between them is a complex dynamic process that is repeated for a long time. Retailers adopt a static expectation method, that is, the price decision of the next period only considers the optimal strategy of the current period, but the use of static expectations requires retailers to fully grasp the market information. In reality, the market information obtained by retailers is often incomplete because obtaining more market information obviously requires more costs. In many cases, due to information distortion and information asymmetry, it is difficult to obtain perfect information without the energy to research the market. Therefore, the use of static expectations overestimates the retailer's ability to predict market prices. At the same time, retailers' pricing processes are not all rational. Therefore, this paper assumes that both traditional offline channel retailers and online direct sales channel retailers adopt bounded rational expectations. This indicates that the retailer's price decision in the next period depends on a local estimate of the current period's marginal utility. If the retailer's marginal utility is positive in the current period, he will increase the price in the next period. This shows that in each pricing period *t*, the retailer will determine the pricing of the period *t* + 1 according to the pricing of its competitors in order to maximize its own utility. The dynamic adjustment process is as follows:

(12) $$\begin{array}{c} p_{i}\left(t+1\right)=\frac{\partial U_{i}\left(p_{1},p_{2}\right)}{\partial p_{i}}-\alpha_{i}p_{i}^{2}\left(t+1\right),i=1,2\text{,} \end{array}$$

where the parameter *a*_*i*_ is the retailer's price adjustment speed. If the retailer can obtain a greater competitive advantage by increasing the price adjustment parameter *a*_*i*_, so as to achieve its own business purpose, he will continue to speed up the price adjustment. We get the discrete dynamics of the price game for a multichannel supply chain:

(13) $$\begin{array}{c} \left\{\begin{array}{c} p_{1}\left(t+1\right)=p_{1}\left(t\right)-\alpha_{1}p_{1}^{2}\left(t+1\right)\left[\left(\frac{a_{1}}{b_{1}}-\frac{c}{p_{1}}\right)+\frac{\varepsilon p_{2}}{\beta \left(c+2p_{2}\right)}\right]\text{,}\\ p_{2}\left(t+1\right)=p_{2}\left(t\right)-\alpha_{2}p_{2}^{2}\left(t+1\right)\left[\left(\frac{a_{1}\varepsilon p_{2}}{b_{1}\beta \left(c+2p_{2}\right)}\right)+\frac{b_{2}}{v\left(c+2p_{2}\right)}\right]\text{,}\\ p_{1}\left(t\right)=p_{1}\left(t\right)-\alpha_{1}p_{1}\left(t\right)\left(\frac{a_{1}}{b_{1}}-\frac{c}{p_{1}}\right)\text{.} \end{array}\right. \end{array}$$

From the perspective of actual competition, the economic significance of the stability of the four equilibrium points of the market is given. The prices of the two retailers are both zero, which means that the two retailers have given up operating their own retail channels and withdrawn from the market, or are operating at a loss. Such a market equilibrium is obviously unstable and even impossible to happen. Both the traditional retail market and the emerging online direct selling channel market have huge potential for development, so no matter which channel a retailer withdraws from the competition, its market share will be completely occupied by other retailers.

## 4. Results and Analysis

### 4.1. Cross-Border M&A of Company A by Company B in the Financial Industry

This article will select a case of cross-border mergers and acquisitions in the financial industry for empirical analysis. Company A in China's financial industry acquired company B in Sweden in 2020. With the final closing ceremony, company A completed the acquisition of the entire equity of company B for US$1.8 billion, and obtained the ownership of company B.

The current status of China's financial industry is as follows: a lack of core technologies, low brand awareness, difficulties in expanding overseas markets, weak team R&D capabilities, and lack of mature global operation experience and mechanisms. This largely explains the motivation of Chinese financial enterprise A to embark on the road of cross-border mergers and acquisitions. Company A's finance is aimed at customers with low- and middle-income levels in China, and the brand's international influence is not enough.

The products produced by company B are mainly for middle- and high-level users. The brand is famous all over the world for luxury, comfort, and safety. Especially in terms of safety, the technical level of company B has been leading the financial industry technology of the whole world. The operation of company B has been hit hard by the financial tsunami, and its cash flow is facing a serious crisis. Affected by the huge decline in purchasing power, the sales volume is also not as good as before. The continuing operation will face the dilemma of the capital chain being cut off, and it is urgent to find a new buyer to survive.

Analyzing the financial statements of company B, it can be found that company B has been in a state of loss, but the degree of loss varies in different periods. The quarterly financial data of company B from 2017 to 2021 (20 quarters) are shown in Figure 3.

In 2018, it decreased by 20% year-on-year, and in 2019, it decreased by 11% year-on-year. It can be seen that the decline in sales volume has become smaller. This situation provides an opportunity for China's financial industry to seek overseas mergers and acquisitions. Before the acquisition, company A was in good financial condition and had a large amount of cash flow, which could fully meet the requirements of the acquisition amount. The cash flow at the end of the accounting year is increasing year by year. Company A's financial situation is running well, and it is in urgent need of external expansion and pursuing a higher level of technology. Company B meets the requirements of company A in terms of technology and brand. The cash flow of company A before the acquisition is shown in Figure 4.

According to statistics, the investment environment of the country where company B is located has been ranked high in the world, and Sweden basically has an open and friendly investment policy. In order to obtain the international investment environment rating of Sweden more accurately, according to the description of the target enterprise investment environment assessment subsystem constructed, the investment environment rating of the country where the company is located is carried out. The evaluation details are shown in Figure 5.

Company A faces many risks, the most important of which are technology integration risks, labor relations handling risks, cultural integration risks, and brand strategy risks. In order to more accurately understand the risks after mergers and acquisitions, it is necessary to evaluate the investment of the companies after mergers and acquisitions and to predict the risks through the evaluation results.

### 4.2. Monte Carlo Simulation of Financial Risk of Cross-Border M&A of Company A

#### 4.2.1. The Basic Data Assumptions of the Simulation Model of Company A's Merger and Acquisition of Company B Are Determined

Investment: The initial investment is based on the acquisition amount of US$1.8 billion; in the future, some additional investment will be made for research and development. Assume that 1 year after the merger, an investment of 10,000 million yuan is required to hire new employees; 3 years after the merger, another 10,000 million yuan is invested to build a new R&D center in Europe. Assuming continuous operation, this simulation simulates the financial data for 10 years after the merger.

The turnover in 2020 of the base year is a random variable that obeys a triangular distribution. If company A can achieve the maximum production capacity in previous years at the initial stage of the merger, the maximum turnover that can be achieved is 30,900 million yuan. If there are many frictions in the initial stage of the merger, it can only meet the minimum production capacity of company A in previous years, and the minimum turnover is 12,900 million yuan. Since the research time has exceeded 2020, it can also be seen from the financial statements of company A in 2020 that the actual turnover of the year is about 20,200 million yuan, and this value is between the historical maximum and minimum values, so the possible value is set at 20200 million yuan. The company spends a lot of energy on personnel integration, corporate culture unification, standardization, etc., and its turnover changes within an average of plus or minus 10% compared with the previous year. Therefore, it is assumed that the annual growth rate of company A's turnover in the 2nd to 3rd years obeys—a random variable uniformly distributed in the interval of 10%. From the 4th year after the merger, the company's production capacity should return to historical levels, with historical 12-year annual turnover growth. According to the law of rate change to assume the range of annual growth rate of turnover of company A from 4 to 10 years after the merger, through the collected financial data of company A's turnover from 1998 to 2019, we calculated the annual growth rate of each year compared with the previous year. The turnover of company A from 2017 to 2021 (20 quarters) is shown in Figure 6.

#### 4.2.2. Calculation Results of a Model Simulation

According to the principle of value selection in the basic data determined by the simulation model, run Crystal Ball software, randomly select random numbers according to the probability distribution determined above, and combine them for calculation. The cross-border investment risk prediction results of the three algorithms are shown in Figure 7.

Through this simulation, the calculation results of an experiment are obtained. The results show that the net present value of the M&A project is 150.616 billion yuan, the internal rate of return has reached 43.54%, and it has a high antirisk ability.

However, one calculation result shows the comprehensive effect of each factor. After random sampling, the repeated calculation is more convincing.

Crystal Ball software facilitates repeated sampling of values and can automatically generate reports on the statistics of predictors.

#### 4.2.3. 1000 Simulated NPV Result Data

Theoretically speaking, the more simulation times, the more correct the result, but the corresponding manpower and material resources are needed to calculate and sort out. Relatively few simulation times will affect the reliability of the simulation results, generally between 200 and 500 times. In order to describe the change in NPV more accurately, 1000 times calculations are set this time. The operation process and value are realized with the help of Crystal Ball software. The cumulative probability that the NPV is greater than or equal to zero is *P* (NPV ≥ 0) = 60%.  Figure 8 shows the time consumption of the three algorithms for cross-border investment risk prediction.

### 4.3. Early Warning Analysis of a Company's Cross-Border M&A

After 1000 simulations, the output results of NPV and IRR are obtained. The cumulative probability of NPV greater than or equal to 0 is *P* (NPV ≥ 0) = 60%, and the cumulative probability of IRR between 30% and 56.67% is 32.59%. The investment environment of the country where company B is located has a score of 90 points, and the investment environment can be rated as excellent with few restrictions on foreign investment, and company B is technology intensive and has a brand advantage. From the cumulative probability histogram of IRR, it can be judged that company A has the weak antirisk ability and is in the financial deterioration range. In this way, it can be concluded that company A has certain financial risks in the 10 years after the acquisition of company B, and the police level is set as a serious warning.

After company A successfully acquires company B, it cannot relax its vigilance. In the face of serious warnings, first of all, it must pay great attention to the integration between companies and control production costs. While growing, the cost of sales should be reduced as much as possible; secondly, to retain the advantages of the B brand and maintain its brand influence in the international market, the production technology of company A should learn from company B to narrow the technological gap. At the same time, it also launched the A product into the international market, thereby expanding its market share.

## 5. Conclusion

In order to solve the problem of too long intermediate transmission time caused by too large intermediate data, a “three-step compression” strategy is proposed to reduce the size of intermediate output data that need to be transmitted. The attention mechanism selects important channels and the third step data quantization operation. In order to meet the application's different preferences and specific requirements for computing delay or inference accuracy, an optimal division point selection algorithm is proposed that comprehensively considers factors such as DNN model layer type, network bandwidth, device computing power, and delay or accuracy requirements. Taking the profit of the system as the evaluation index, the influence of the chaos phenomenon on the operating efficiency of the system is evaluated. We found that the system with the highest efficiency (maximum profit) is when the competitive price of the two retailers is stable at the Nash equilibrium point, and when the system is in a cycle bifurcation or chaotic state, a very small change in price may cause a relatively small change in the market evolution behavior. Therefore, in order to avoid the loss of the system and the profits of each retailer, retailers should be more cautious and scientific when setting prices, especially when the market is chaotic due to free competition, timely analysis of information, and using certain chaos control methods are very necessary. Based on the discounted cash flow model, the postmerger alarm forecasting subsystem uses Monte Carlo simulation for each variable risk factor to examine the comprehensive impact of various risk factors on the net present value. It is implemented with the help of Crystal Ball software. The cumulative probability that the net present value of the later *t* years is greater than zero; the alertness interval is divided into two dimensions, the investment environment evaluation and the alertness prediction value of the subsystem, to jointly judge the alertness interval after the merger and divide the alertness into five levels: giant police, heavy police, medium police, light police, and no police. This paper selects company A in the financial industry to acquire company B in Sweden and synthesizes the investment environment rating of the country where company B is located and the cash flow of company A after the merger.

## Figures and Tables

**Figure 1:** ECCI overall architecture.

**Figure 2:** “Three-step compression” strategy.

**Figure 3:** Quarterly financial data of company B from 2017 to 2021 (20 quarters).

**Figure 4:** Company A's cash flow before M&A.

**Figure 5:** Investment climate rating of the country where company B is located.

**Figure 6:** Company A's turnover from 2017 to 2021 (20 quarters).

**Figure 7:** Cross-border investment risk prediction results of three algorithms.

**Figure 8:** Time consumption of cross-border investment risk prediction by three algorithms.

## Data Availability

The data used to support the findings of this study are included within the article.
